The article "Analysis of Spatial Distribution of CVD and Multiple Environmental Factors in Urban Residents" was published in 2022. Journal: Comput Intell Neurosci.

# Analysis of Spatial Distribution of CVD and Multiple Environmental Factors in Urban Residents

**DOI:** 10.1155/2022/9799054

**Published:** 2022-03-16

**Authors:** Beichen Wang, Kangkang Gu, Dong Dong, Yunhao Fang, Lingling Tang

**Affiliations:** ^1^School of Architecture & Planning, Anhui Jianzhu University, Hefei, Anhui 230022, China; ^2^School of Architecture and Urban Planning, Huazhong University of Science and Technology, Wuhan, Hubei 430000, China; ^3^College of Architecture and Art, Hefei University of Technology, Hefei, Anhui 230009, China

## Abstract

Cardiovascular disease (CVD) poses a serious threat to urban health with the development of urbanization. There are multifaceted and comprehensive influencing factors for CVD, so clarifying the spatial distribution characteristics of CVD and multiple environmental influencing factors is conducive to improving the active health intervention of urban environment and promoting the sustainable development of cities The spatial distribution characteristics of CVD deaths in a certain district, Bengbu City, Huaihe River Basin, China, in 2019 were explored, and the correlation between multiple environmental factors and CVD mortality was investigated in this study, to reveal the action mechanism of multiple environmental factors affecting the risk of mortality. Relevant studies have shown that (1) CVD deaths are characterized as follows: male deaths are more than females; the mortality is higher in those of higher age; most of them are unemployed; cardiocerebral infarction is the main cause of death; and the deaths are mainly distributed in the central city and near the old urban area. (2) The increased CVD mortality can be attributed to the increased density of restaurants and cigarette and wine shops around the residential area, the increased traffic volume, the dense residential and spatial forms, the low green space coverage, and the distance from rivers. Therefore, appropriate urban planning and policies can improve the active health interventions in cities and reduce CVD mortality.

## 1. Introduction

A great number of studies have demonstrated the high mortality and disability rate of cardiovascular disease (CVD) [1] and the resulting global burden of diseases [2]. The traditional risk factors for CVD include hypertension, diabetes, dyslipidemia, obesity, smoking, alcohol consumption, and lack of physical exercise. However, under the biological-psychosocial medical model, the influencing factors on health are multifaceted and comprehensive, including environmental factors. Previous studies have shown that the urban population is more likely to suffer from cardiovascular diseases than the rural population in some developing countries [3]. Industrialization, urbanization, aging, and constant changes in the ecological environment and lifestyle have brought challenges to people's health in the rapid urban development. A lot of cities are experiencing a major shift in the disease spectrum from infectious diseases to chronic noncommunicable diseases. Therefore, it is conducive to improving active health interventions in urban environment and promoting sustainable urban development in the future to identify the mortality distribution characteristics of CVD and environmental influencing factors.

Previous studies have shown that unreasonable diet, excessive oil, and salt intake will increase the pressure of human circulatory system [4], thereby leading to CVD morbidity and mortality. The increase in the amount of physical activity, such as work, commuting, and leisure, will appropriately reduce the risk of CVD-related death [5], and the accessibility of sports and leisure activity facilities and open space will also have an influence on the level of physical activity of residents [6]. Residents will tend to commute by non-motor vehicles and increase daily activities provided that the urban road slow traffic system is perfect and the bus stops are dense [7]. In addition, residents engaged in manual work will have increased daily activities [8], thus reducing the risk of death. Air pollution [9–11] and noise pollution [12] constitute the important risk factors for CVD, of which long-term air pollution has a greater impact on CVD than short-term one [13]. The closer distance to the pollution source or the greater density of the surrounding pollution sources will increase the possibility of exposure to pollutants [14, 15], including a large number of industrial pollutants [16], the cooking fumes from [17], the exhaust gas emissions of motor vehicles, and urban transportation facilities, such as railways, subway lines, and airports [18]. Roads and restaurants produce noise pollution while causing air pollution, thereby leading to the occurrence of cardiovascular diseases [19]. The nearer distance from rivers and the higher green space coverage can effectively reduce the concentration of particulate matter (Douglas, W., and [20–22]) and lower CVD mortality. Cold weather and sudden temperature drop in winter are prone to causing overreaction of human function, resulting in death from acute CVD [23, 24]. The difference in temperature in different urban regions will lead to the difference in mortality.

In general, current studies focus on the macro-level of county [25], prefecture [26], and state [25], but neglect the small scales, such as communities and streets; meanwhile, the consideration of environmental factors is relatively simple, and the influence of aging population and old urban areas is relatively ignored. A large number of people in the Huaihe River Basin in Central China died of chronic diseases caused by the environment many years ago [27]. The urban environmental pollution is relatively serious now, seriously endangering the physical and mental health of residents. In view of this, the distribution characteristics of CVD deaths were analyzed, and the influences of multiple environmental factors on CVD were systematically investigated in this study with the old urban area in Bengbu City of Huaihe River Basin as the subject, to reduce CVD mortality by proper urban planning and policies, and provide certain research ideas for healthy city construction in other areas of Huaihe River Basin.

## 2. Materials and Methods

### 2.1. Study Area

Bengbu City, located in the south of Huaihe River Basin, China, is characterized by high population density and rapid urbanization [28]. Bengbu was an important industrial city and traffic hub in China before, where a large number of chemical, pharmaceutical, and building materials enterprises and the heavy traffic pressure have produced a large amount of pollution in Bengbu, seriously affecting the physical and mental health of residents. A certain district is located in the Western old urban area of Bengbu City, adjacent to the commercial and cultural center of the city in the east and the Huaihe River (one of the seven major rivers in China) in the north, and it is also the administrative area with the largest population in Bengbu City, so it is suitable for the research on urban environment and population health. The study area consisted of 12 blocks numbered YH01-YH12 in a certain district, which were divided into 2,744 spatial units by 100 m grid (Figure 1). The study area is located in the mid-latitude region, where northeasterly wind is the most prevalent throughout the year, the average temperature in January is 1°C, and it is susceptible to cold waves in winter.

### 2.2. Data Sources

#### 2.2.1. Sources of Data Related to CVD

The data of cardiovascular disease (CVD) mortality were collected from the population whose cause of death was cardiovascular disease (ICD-10 code I00-I99) determined by Bengbu Health Commission in 2019, including detailed address, age, gender, and occupation before death. Inpatients whose home addresses and affiliations were not within the study area were excluded, so the final number was 469 in total. The number of resident population in a certain district in 2019 was derived from the official bulletin of Bengbu National Bureau of Statistics.

#### 2.2.2. Environmental Data Sources

The land use data and built environment data in environmental data were obtained from the Anhui Urban & Rural Planning and Design Institute, and the data contained the main uses of each land in a certain district in 2019, as shown in Figure 2(a), which included roads, green space and river, residential land, industrial land according to urban land classification, and the base area and floor number of each building. Commercial and bus stops are derived from open-source point-of-interest (POI) data, which are characterized by large sample size, wide coverage, and detailed spatial resolution, making spatial analysis more comprehensive, objective, and in-depth, as shown in Figure 2(b). Data of environmental pollution indexes were obtained from the Bengbu Bureau of Ecology and Environment, and the pollution values of each spatial unit were obtained by the interpolation method for the pollution monitoring point data. Data of land surface temperature and vegetation coverage were derived from Landsat 8 remote sensing data in January 2019 provided by USGS and coded LC81210372019023LGN00.

### 2.3. Influencing Factor Index System

To explore the distribution characteristics of cardiovascular disease (CVD) and environmental influencing factors in urban residents, the basic characteristics and spatial distribution characteristics of CVD deaths were analyzed, and the correlation between various environmental influencing factors and CVD mortality was explored (Figure 3). Environmental influencing factors included land use, road traffic, spatial form, and natural environment, with their potential impacts on CVD shown in Table 1. The calculation formula for CVD mortality is as follows:

(1) $$\begin{array}{c} \text{Mortality}=\;\frac{\text{Nc}}{\text{Np}}\times 100\text{\%,} \end{array}$$

where Nc is the number of deaths due to CVD in a unit and Np is the total population in a unit.

### 2.4. Study Methods

#### 2.4.1. Spatial Autocorrelation Assessment

Global spatial autocorrelation [29] is usually measured by Moran's *I*, and the aggregation of subregional geospatial CVD deaths is judged according to the spatial distribution pattern of the whole region. Moran's *I* range is [−1, 1], and the larger value indicates the more obvious spatial correlation, and the smaller value indicates the greater spatial difference, with the specific calculation formula as follows:

(2) $$\begin{array}{c} \text{Moran's }I=\frac{n\sum_{i=1}^{n}\sum_{j=1}^{n}w_{ij}\left(x_{i}-\bar{x}\right)\left(x_{j}-\bar{x}\right)}{\sum_{i=1}^{n}w_{ij}\sum_{j=1}^{n}\sum_{i=1}^{n}{\left(x_{i}-\bar{x}\right)}^{2}}\left(i\neq j\right), \end{array}$$

where *n* is the number of study units; *x*_*i*_ and *x*_*j*_ represent the CVD mortality in area *i* and area *j*, respectively. ‾*x* represents the average CVD mortality; *W*_*ij*_ represents the spatial weight matrix.

Local spatial autocorrelation [30] can reveal the heterogeneity of local space, make up for the atypical characteristics of local areas in the whole region, and fully reflect the variation trend of local geospatial epidemic risk. The spatial difference in CVD mortality was measured by local indicators of spatial association (LISA) in this study, with the calculation formula shown as follows:

(3) $$\begin{array}{c} {\text{LISA}}_{i}=z_{i}\sum_{j}w_{ij}z_{j}\text{,} \end{array}$$

where *z*_*i*_ and *z*_*j*_ represent the standardized values of CVD mortality in area *i* and area *j*, respectively. *W*_*ij*_ represents the spatial weight matrix. In the LISA of local spatial autocorrelation, CVD mortality can be divided into four categories: high-high clustering (H-H), high-value clustering; low-low clustering (L-L), low-value clustering; high-low clustering (H-L), outliers with high values mainly surrounded by low values; and low-high clustering (L-H), outliers with low values mainly surrounded by high values.

#### 2.4.2. Spearman's Rank Correlation

To investigate the relationship between CVD and environmental factors, the correlation between the mortality rate of CVD (dependent variable) and the values of various environmental factors (independent variables) was comprehensively measured by Spearman's rank correlation [31], with the specific formula referred to formula (3). Compared with Pearson's correlation, Spearman's rank correlation can make up for the fact that the correlation of environmental factor values may not be linear and are interfered with detection error and other factors, thus making the correlation more significant [32]. CVD mortality and environmental factor values were subject to normalized processing (value range of [0, 1]), which was used to balance the dimensional gap of data and enable different data to be counted under the same conditions.

(4) $$\begin{array}{c} \rho =1-\frac{6\sum_{i=1}^{n}d_{i}^{2}}{n\left(n^{2}-1\right)}, \end{array}$$

where *ρ* is Spearman's correlation coefficient, with the value range of [−1, 1], and the larger absolute value indicates the stronger correlation. *n* represents the number of areas of CVD mortality, and *d*_*i*_ represents the rank difference between dependent variable (CVD mortality) and independent variable (environmental influencing factor values).

## 3. Results

### 3.1. Basic Characteristics of CVD Deaths

A total of 469 people died of cardiovascular disease (CVD) in the study area in 2019 according to the statistics of collected death data, with the basic characteristics of death population, such as gender, age, occupation, death season, and specific diseases leading to death, shown in Table 2.

The analysis results showed that the mortality among male CVD patients was significantly higher than female patients, with a ratio of about 1.18 : 1. The elderly over 80 years accounted for 54.15% of CVD deaths, and those under 60 years only accounted for about 10%, indicating that the higher the age, the higher the mortality. Winter (December to February of the following year) and autumn (September to November) were the most frequent periods of CVD deaths, accounting for 27.93% and 27.72% of the total number of deaths, respectively, and the mortality in autumn and winter was 1.25 times higher than that in spring and summer. The largest number of CVD deaths was among the unemployed (26.01%), followed by workers (6.61%), freelancers (5.54%), and farmers (2.56%). Among the specific diseases causing death, cerebral infarction and myocardial infarction accounted for 24.09% and 19.62%, followed by coronary heart disease (17.70%).

### 3.2. Spatial Distribution of CVD Deaths

In 2019, there was a significant difference in the number of CVD deaths among different units in the study area. YH07 and YH08 accounted for 73.56% in terms of deaths, of which YH08 had the largest number of CVD deaths, namely 180, followed by 165 deaths in YH07 and no deaths in YH10 and YH11. The kernel density analysis of CVD deaths was conducted with ArcGIS software (Figure 4), and unit density of CVD deaths in the study area could be calculated, which could intuitively reflect the distribution of CVD deaths in a continuous area [33]. The analysis results suggested that CVD deaths were mainly distributed in the vicinity of Unit YH09 in Zhanggongshan Park and the north of Unit YH08 near the Huaihe River. The area near YH09 was an old urban area of Bengbu, characterized by high population density and serious aging. A total of 365 people died within the 1 km buffer zone of Zhanggongshan Park, accounting for 77.82% of the total deaths; moreover, the density of deaths was lower in the area farther away from Zhanggongshan Park. The north of YH08 is also a large population gathering area, close to the central city of Bengbu and Huaihe River in the east.

Among 2,744 study units, 1,053 units containing residential land (i.e., unit population greater than 0) were taken as the research samples after the outlier samples were excluded. The normalized mean value of the calculated CVD mortality values of all study units was normalized to be 0.008, with the standard deviation of 0.055, indicating that there were significant spatial differences in the CVD mortality. Global Moran's *I* index analysis showed that the spatial distribution of normalized mortality index was of spatial autocorrelation (Moran's *I* > 0, *Z* = 2.192, *P* < 0.05), indicating that there was a significant spatial aggregation phenomenon in the distribution of CVD deaths. In addition, there was a local spatial autocorrelation in the normalized mortality index according to the spatial distribution of LISA clustering (Figure 5), in which H-H clustering (22) was mainly distributed in the middle of YH08, forming a significant H-H clustering of CVD mortality. L-L clusters (121) were mainly distributed in YH05, YH10, and YH12, with a few scattered clusters in other units, showing more L-L clusters in the CVD mortality.

### 3.3. Relationship between Environmental Factors and CVD Mortality

The results of Spearman's rank correlation analysis are shown in Table 3. Among land use, road traffic, spatial form, and natural environment, there are 14 environmental factors showing significant correlation and statistical significance with CVD mortality (*P* < 0.05). There was no correlation between industry and CVD mortality (*P* > 0.05). The spatial distribution of environmental influencing factors is shown in Figure 6.

#### 3.3.1. Land Use

The model showed that the residential density was positively correlated with the CVD mortality (*ρ* = 0.127), indicating that the higher the residential density, the higher the CVD mortality. The density of fast-food restaurants and the density of cigarette and wine shops showed a significant positive correlation with the CVD mortality in the 500 m buffer zone (*ρ* = 0.287, *ρ* = 0.286), indicating that the higher the density of fast-food restaurants and cigarette and wine shops, the higher the mortality. There was a significant negative correlation between the nearest distance to the open space and the CVD mortality (*ρ* = −0.189), indicating that the farther from the park, the lower the CVD mortality. The normalized difference vegetation index (NDVI) in January showed a significant negative correlation with CVD mortality (*ρ* = −0.179), indicating that the higher the vegetation coverage, the lower the CVD mortality.

#### 3.3.2. Road Traffic

The model showed that the road network density and the intersections within the 500 m buffer zone were significantly positively correlated with the CVD mortality (*ρ* = 0.138, *ρ* = 0.220), indicating that the greater the traffic volume, the higher the CVD mortality. Meanwhile, there was a significant positive correlation between the density of bus stops and the CVD mortality within the 500 m buffer zone (*ρ* = 0.238), indicating that there was a lower risk of death among the people living in the area with sparse bus stops.

#### 3.3.3. Spatial Form

The model showed that building density and floor area ratio were significantly positively correlated with CVD mortality, with the correlation coefficients of 0.104 and 0.115, indicating that high-density space would increase the CVD mortality.

#### 3.3.4. Natural Environment

There was a significant positive correlation between the distance to the nearest river and the CVD mortality (*ρ* = 0.121), indicating that the closer to the river, the lower the CVD mortality. The average annual PM_2.5_ and PM_10_ were significantly positively correlated with the CVD mortality, with the correlation coefficients of 0.088 and 0.072, indicating that the higher the average annual particulate matter (PM) concentration, the higher the CVD mortality. The average temperature was negatively correlated with the CVD mortality, with a correlation coefficient of -0.135, indicating that the lower the temperature in winter would contribute to the increase in the CVD mortality.

## 4. Discussion

1. The characteristics of CVD deaths were significant and of spatial clustering.
2. Consistent with the conclusions of previous international statistical studies, the CVD deaths were characterized as follows: male deaths were more than females; the mortality is higher in those of higher age; most of them are unemployed; and cardiocerebral infarction was the main cause of death. In addition, the deaths were mainly distributed in the old urban area, and there was a significant spatial clustering phenomenon [34]. Previous studies have shown that alcohol abuse [35] and smoking [36] can affect the cardiovascular system, and males are more likely to do alcohol abuse and smoking than females, causing the difference in mortality. The risk of cardiac arteriosclerosis will increase with age; that is, the mortality is higher in those of higher age [37]. Working can reduce the risk of CVD [8], and the risk of CVD is lower in residents engaged in manual work, but higher in those unemployed. Low temperature and sudden drop in air temperature will cause vasoconstriction and elevated blood pressure of human body, increasing the risk of sudden myocardial infarction [23, 24]; therefore, autumn and winter are the seasons of high incidence of CVD, and the mortality is higher in the urban areas with lower urban temperature [38].
3. The higher density of restaurants and cigarette and wine shops will increase the CVD mortality.
4. It has been further confirmed in this study that the density of restaurants and smoking restaurants around the residential area showed a significant positive correlation with the CVD mortality. The daily activity distance that can meet the basic material and life needs of residents by 10-min walking is 500 m [39]. Handy et al. [40] found that the frequency of walking to businesses was positively correlated with the number of businesses within the service radius; therefore, people in the areas with highly dense restaurants and cigarette and wine shop will have higher probability of dining out and buying cigarettes and wines. In the study area, located in northern Anhui, the restaurant diet contains high fat and salt, and the dense dining facilities will bring more cooking fumes, sewage, and other environmental pollution, in which a lot of fat and cholesterol oxide [17]will lead to hypertension, hyperlipidemia, and other metabolic disorder CVD, and the increased probability of buying alcohol and tobacco will raise the risk of alcoholism, thereby causing sudden death [17].
5. The influence of environmental factors related to particulate matter concentration on the CVD mortality.
6. Consistent with the conclusion of previous studies abroad, long-term exposure to high levels of pollutants will affect the human circulatory system [41], thereby inducing CVD mortality. According to the data of disease burden from Barcelona, Spain, it was estimated that 849 cases of CVD could be prevented each year if the exposure level of air pollution could be reduced to the WHO recommended level [42]. There is a higher risk of death for residents in areas with high concentrations of particulate matter. The finding is further confirmed in this study: the increased traffic volume [43], dense bus stops [44], and dense residential and spatial forms [45, 46], low green space coverage [47], and longer distance from rivers [47] can increase the CVD mortality, of which the possible reason may be associated with the increased concentration of local particulate matter and other noise pollution and psychological harm.
7. Discussion on the correlation between industrial and open activity space and CVD mortality.
8. Different from general studies, it is found that there is no significant relationship between CVD mortality and industry in this study, for which reason may lie in that northeasterly wind is the most prevalent in the study area throughout the year, and there are few residential areas located downwind of industry, only accounting for less than 10% of the study units; therefore, the influence of industry on the study unit is not significant. Meanwhile, this study also reveals that CVD mortality is lower in the areas farther from open space area, and the possible reason is that the study area is an old urban area that lacks green space, there are only 3 parks with the area of more than 1 ha within or 500 m from the study area (aggregated distribution), and there is relatively little activity space, which also is the common fault of an old urban area. The elderly are at high risk of dying from CVD, and they will deliberately choose the area around the open activity space when choosing housing, which will have a certain impact on the conclusion.

## 5. Conclusions and Prospects

To explore the distribution characteristics of cardiovascular disease (CVD) in urban residents and the environmental influencing factors, this study analyzed the basic characteristics and spatial distribution characteristics of CVD death population, explored the correlation between multiple environmental factors and CVD mortality, and revealed the factors affecting the risk of death and its mechanism, with the main conclusions as follows:

1. The correlation study conducted in this study is of good scientific nature and research significance, and the conclusions are consistent with international studies. Therefore, the study methods can provide some research ideas for the construction of healthy cities in the Huaihe River Basin or other regions.
2. With obvious characteristics, CVD deaths are mainly distributed in the vicinity of Unit YH09 in Zhanggongshan Park and the north of Unit YH08 near the Huaihe River. Therefore, attention should be paid to the key areas with the maximum number of CVD deaths and the population at high risk, and medical input should be increased to reduce the death risk.
3. Because long-term exposure to high pollutants in the environment will cause CVD death, the following measures can be taken to reduce the CVD mortality in the construction of healthy cities in the future: increase traffic arterial roads around residential areas to reduce the traffic volume and vehicle exhaust emissions in residential areas; increase open space to reduce living and spatial density; plant more plants and building more rivers to reduce the local air pollution; and make dispersed layout of commercial facilities, such as restaurants and cigarette and wine shops, around residential areas to effectively reduce the risk of CVD death. Meanwhile, attention should also be paid to the influence of the areas with a higher density of the elderly on the analysis results.

Appropriate urban planning and policies can improve the active health interventions in cities and reduce the CVD mortality. To a certain extent, it can also provide more research perspectives for the construction of healthy cities in the future, and promote the development of healthy cities. In addition, this study is based on panel data, and little consideration is given to the changes of built environment and CVD mortality caused by time changes, so time series related research will be carried out in the future. At the same time, different lifestyles will affect CVD mortality, so further research on the correlation between residents' lifestyles and CVD mortality will be conducted in the future.

## Figures and Tables

**Figure 1:** Area bitmap.

**Figure 2:** Present distribution.

**Figure 3:** Conceptual framework.

**Figure 4:** Distribution map of CVD death population.

**Figure 5:** Spatial autocorrelation distribution of CVD normalized mortality index.

**Figure 6:** Spatial distribution of environmental influencing factors.

**Table 1:** Environmental influencing factors.

Category	Subcategory	Variable	Unit	Definition	Potential impact of hypothesis
Land use	Live	Residential density	%	Living area/total land area	Cause pollution and physical and mental stress
	Industry	Distance from the nearest industry	m	Distance from the nearest industry	The closer you are to industry, the more pollution you get
	Business	Fast-food restaurant density	Pcs/ha	Number of fast-food restaurants in 500 m buffer zone/buffer zone area	Intake relatively high salt and oil
		Tobacco and liquor shop density	Pcs/ha	Number of tobacco and liquor stores in 500 m buffer zone/buffer zone area	Increase the risk of alcohol and smoking
	Open the activity space	Distance from the nearest open space	m	Distance from the nearest open space	It is more convenient to exercise and relax
	Vegetation cover	Normalized difference vegetation index (NDVI)	—	NDVI in 2019	Vegetation coverage can reduce air pollution, increase green vision rate, and delight body and mind
Road transport	Traffic	Road network density	m/ha	Road length/total land area	Increase air and noise pollution
	Road intersection	Road intersection density	Pcs/ha	Number of road intersections in 500 m buffer zone/buffer zone area	More air and noise pollution
	Bus stop	Bus stop density	Pcs/ha	Number of bus stops in 500 m buffer zone/buffer zone area	It is more convenient to travel and increase the amount of activities
Spatial form	Building density	Building coverage	%	Total area of building basement/total area of land	High density reduces the wind speed, which increases the concentration of air pollutants and makes people depressed
	Volume fraction	Volume fraction	—	Total construction area/total land area	High density reduces the wind speed, which increases the concentration of air pollutants and makes people depressed
Natural environment	River	Distance from the nearest river	m	Distance from the nearest river	Adsorption of air particles by water body
	Particulate matter (PM)	Mean PM_2.5_	Ug/m^3^	Average PM_2.5_ in 2019	Increase air pollution
		Mean PM_10_	Ug/m^3^	Average PM_10_ in 2019	Increase air pollution
	(Ground) surface temperature	Mean surface temperature	°C	Surface temperature in January 2019	Cold winter temperatures increase the risk of death

**Table 2:** Statistics of CVD death population.

Category	Classify	Death toll	Proportion of deaths (%)
Gender	Man	254	54.16
	Woman	215	45.84
Age	≥80 years old	254	54.15
	70–79 years old	109	23.24
	60–69 years	58	12.37
	<60 years old	48	10.23
Occupation	Unemployed	122	26.01
	Worker	31	6.61
	Individual operator	26	5.54
	Farmer	12	2.56
	Other	278	59.27
Dead season	Spring (March–May)	110	23.45
	Summer (June–August)	98	20.90
	Autumn (September–November)	130	27.72
	Winter (December–February of the following year)	131	27.93
Specific diseases leading to death	Cerebral infarction	113	24.09
	Cardiac infarction	92	19.62
	Coronary heart disease	83	17.70
	Encephalorrhagia	55	11.73
	Pulmonary heart disease	43	9.17
	Other	83	17.70

**Table 3:** Correlation between environmental factors and CVD mortality.

Category	Subcategory	Variable	Ρ (correlation coefficient)	*P* value (double side)
Land use	Live	Residential density	0.127^*∗*^	0.000
	Business	Density of fast-food restaurants in 500 m buffer zone	0.287^*∗∗*^	0.000
		Density of tobacco and liquor stores in 500 m buffer zone	0.286^*∗∗*^	0.000
	Industry	Distance from the nearest industry	-0.011	0.717
	Open the activity space	Distance from the nearest open space	−0.189^*∗∗*^	0.000
	Vegetation cover	Normalized difference vegetation index (NDVI)	−0.179^*∗∗*^	0.000
Road transport	Traffic	Road network density	0.138^*∗∗*^	0.000
		Road intersection density in 500 m buffer zone	0.220^*∗∗*^	0.000
	Bus stop	Density of bus stops in 500 m buffer zone	0.238^*∗∗*^	0.000
Spatial form	Building density	Building coverage	0.104^*∗∗*^	0.001
	Volume fraction	Volume fraction	0.115^*∗∗*^	0.000
Natural environment	River	Distance from the nearest river	0.121^*∗∗*^	0.000
	Particulate matter (pm)	Average annual pm_2.5_	0.088^*∗∗*^	0.004
		Average annual pm_10_	0.072^*∗*^	0.020
	(Ground) surface temperature	Surface temperature in January 2019	−0.135^*∗*^	0.000

^*∗*^ *P* < 0.05, ^*∗∗*^*P* < 0.01.

## Data Availability

The datasets used during this study are available from the corresponding author on reasonable request.
